# Comparison of the Ameliorating Effects of Valsartan and Amlodipine on Vascular Endothelial Dysfunction and Oxidative Stress in Elderly Patients with Type H Hypertension

This article has been retracted.

**DOI:** 10.1155/2022/5054511

**Published:** 2022-08-08

**Authors:** Lijuan Zhang, Hua Yang, Ping Yang

**Affiliations:** Department of Geriatrics, The First People's Hospital of Lianyungang, Lianyungang, Jiangsu, 222000, China

## Abstract

**Objective:**

To explore whether long-term administration of valsartan or amlodipine can improve vascular endothelial function and reduce the production of reactive oxygen species in patients with H-type hypertension, so as to provide a reference for clinical treatment.

**Methods:**

A total of 82 elderly patients with type H hypertension who were admitted to our hospital from March to August 2017 were selected as the research subjects. The study included a 4-week continuous irrigation period followed by a 24-week randomized treatment period. Forty patients in the valsartan group and 42 in the amlodipine group were treated with 5 mg amlodipine or 80 mg valsartan for 24 weeks. Clinical efficacy, 24 h mean DBP, SBP, and 24HSBP, DBP coefficient of variation, cardiac fatty acid-binding protein (H-FABP), vascular pseudohemophilia factor (VWF), nitric oxide (NO), endothelium-dependent vasodilation function (FMD), nonendothelium-dependent vasodilation function (NMD), malondialdehyde (MDA), GSH-Px, and SOD levels were observed.

**Results:**

The total effective rate was 80.0% (32/40) in the valsartan group and 85.71% (36/42) in the amlodipine group, and the difference was not statistically significant (*P* > 0.05). After 24 weeks of treatment, the 24 h mean SBP, SDP, 24HSBP, and DBP variation coefficients of the two groups were significantly decreased, and there was no statistical significance between the two groups (*P* > 0.05). After treatment, the values of H-FABP, VWF, NO, and MDA in both groups decreased compared with before treatment, while the values of FMD%, NMD%, SOD, and GSH-Px increased compared with before treatment (*P* > 0.05), and the levels of H-FABP, VWF, and NO in the valsartan group were lower than those in the amlodipine group. Meanwhile, FMD%, NMD%, SOD, and GSH-Px levels were higher than those in the amlodipine group (*P* > 0.05).

**Conclusion:**

Valsartan and amlodipine reduce blood pressure, improve vascular endothelial function, and inhibit oxidative stress in elderly patients with H-type hypertension on average. However, valsartan has a better effect on vascular endothelial dysfunction and oxidative stress in elderly patients with H-type hypertension.

## 1. Introduction

Hypertension is one of the serious health problems in China. Endothelial dysfunction is a critical pathological basis for the early phase of hypertension, which leads to hypertensive vascular disease. The mechanism of endothelial dysfunction is complex and closely related to the massive generation of reactive oxygen species (ROS) in the vascular wall. Some in vivo studies have confirmed that antihypertensive drugs correct blood pressure by inhibiting vascular oxidative stress, thereby protecting vascular endothelial cells. Homocysteine (Hcy) is an important intermediate product of the methionine metabolism. Compared with isolated hypertension, hypertension with elevated plasma homocysteine, namely, H-type hypertension, will further aggravate vascular oxidative stress. Valsartan, an angiotensin II receptor blocker (ARB), and amlodipine, a long-acting dihydropyridine calcium channel blocker, are both widely used in the treatment of H-type hypertension. At present, the effect of antihypertensive drugs on vascular endothelial function has been clinically studied in a small population. However, few scholars have paid attention to the effects of valsartan and amlodipine on the function of vascular endothelial cells in patients with H-type hypertension and their antihypertensive effects. The purpose of this study was to investigate whether long-term administration of valsartan or amlodipine in H-type hypertension patients could improve vascular endothelial function and reduce the production of reactive oxygen species.

## 2. Materials and Methods

### 2.1. Research Objects

This study is a prospective randomized controlled trial, and the study protocol was approved by the institutional review board of our hospital. All patients provided written consent. Inclusion criteria were as follows: aged over 60 years old, diastolic blood pressure (DBP) ≥90 mmg or systolic blood pressure (SBP) ≥140 mmg, and plasma Hcy level ≥10 *µ*mol/L. Exclusion criteria were as follows: (1) refractory hypertension, symptomatic hypotension, hypertrophic, or restrictive cardiomyopathy, constrictive pericarditis, acute and chronic cerebrovascular disease, secondary hypertension, hypercalcemia, pregnancy, and chronic liver or renal insufficiency; (2) those with a history of ARB or amlodipine intolerance; (3) patients with cerebral infarction or coronary revascularization within 6 months; and (4) those who have been diagnosed with malignant tumor within 3 years and plan to undergo major surgery during the trial. The sample size was estimated according to the Kadam and Bhalerao method, and based on the above inclusion and exclusion criteria, we selected a total of 82 elderly H-type hypertension patients admitted to our hospital from March to August 2017 as the research subjects, aged ≥60 years. Among them, 50 were males and 32 were females, aged 60–89 years. The mean age was 70.32 ± 6.96 years, and the mean plasma Hcy level was 18.64 ± 6.39 *μ*mol/L. The study consisted of a continuous washout period of 4 weeks followed by a randomized treatment period of 24 weeks. Based on an average of 6 consecutive blood pressure readings at both visits and 24-hour ambulatory blood pressure values at the end of the flushing period, they were randomly assigned to receive 5 mg of amlodipine or 80 mg of valsartan for 24 weeks if they met the inclusion criteria. Finally, 40 patients were included in the valsartan group, and 42 patients were included in the amlodipine group. The age, gender, average course of the disease, plasma Hcy level, and other data of the two groups of patients were basically the same, and there was no statistical difference (*P* > 0.05), which was comparable, as given in Table 1.

### 2.2. Treatment

The patients in both groups were given conventional antihypertensive therapy, and the patients in the valsartan group were given valsartan tablets (Beijing Novartis Pharmaceuticals Co., Ltd., approved by H20173015), with an initial dose of 80 mg/time, once a day. The patients in the amlodipine group were given amlodipine besylate tablets (manufactured by Pfizer Pharmaceuticals Co., Ltd., approved by the State Drug Administration No. H10950224), 5 mg/time, 1 time/d. Both groups were treated continuously for six months. Study medication was provided free of charge throughout the study period. Patients take the study medication between 6 : 00 a.m. and 08 : 00 a.m. every morning before breakfast, except after blood pressure was measured on the day of the clinic and ambulatory blood pressure monitoring was started. Blood pressure was measured at baseline, 8 weeks, 16 weeks, and 24 weeks of treatment. DBP and SBP were measured after sitting for 10 min, and the average value was recorded. If blood pressure did not reach SBP <130 mmHg or DBP <80 mmHg at 8 weeks of treatment, the dose of each drug was doubled. If the blood pressure of both groups did not reach the target blood pressure (SBP <130 mmHg or DBP <80 mmHg) at 16 weeks, an additional 12.5 mg of hydrochlorothiazide was administered, as it has previously been shown to have no effect on oxidative stress. After 24 weeks of treatment with each drug, blood and urine samples were taken in the morning following an overnight fast.

### 2.3. Observation Indicators

#### 2.3.1. Clinical Data Collection and Blood Pressure Measurement

Blood pressure was measured using a noninvasive ambulatory blood pressure monitor (Model 6100). The 24 h mean systolic and diastolic blood pressure were calculated by computer. Before treatment and after 24 weeks of treatment, 3 mL and 4 mL of fasting peripheral venous blood were collected, placed in a heparin anticoagulant tube and a blood collection tube without anticoagulant, respectively, and centrifuged at 4000 r/min for 5 min to separate plasma; serum was separated by centrifugation at 3000 r/min for 15 min. The plasma Hcy concentration was determined by the Siemens Advia2400 automatic biochemical analyzer and the circulating enzyme method. Other relevant demographic, clinical, and laboratory data were collected.

#### 2.3.2. Vascular Endothelial Function Related Indicators

Serum heart type fatty acid-binding protein (H-FABP) and von Willebrand factor (vWF) were determined by enzyme-linked immunosorbent assay (ELISA). The serum NO level was detected by the nitrate reductase method, and the kit was purchased from Shanghai Enzyme Link Biotechnology Co., Ltd. Strictly follow the kit instructions.

#### 2.3.3. Flow-Mediated Dilatation (FMD)

Using the Toshiba Power Vision 8000 high-frequency ultrasound instrument (11 MHz linear array transducer), the right brachial artery FMD was measured. An inflatable tourniquet was placed on the forearm to make the surrounding pressure exceed the systolic blood pressure by more than 50 mmHg for 5 minutes, and then, the cuff was quickly relaxed, and the blood flow velocity was measured by the Doppler echo method. After a 15 min rest, nitroglycerin (400 *µ*g) was administered, and the inner diameter of the right brachial artery (D2) was recorded again. FMD%=(D1−D0)/D0×100%. Nitroglycerin-mediated nonendothelial relaxation function (nitroglycerin-mediated dilation, NMD)% = (D2−D0)/D0 × 100%. All ultrasound examinations were performed by an experienced sonographer operator with a coefficient of variation of 0.79 ± 0.23%.

#### 2.3.4. Oxidative Stress Indicators

In both groups, fluorescence spectrophotometry was used to determine malondialdehyde (MDA), and the thiobarbituric acid method was used to determine glutathione peroxidase (GSH-Px), using the pyrogallol auto-oxidation method to determine plasma superoxide dismutase (superoxide dismutase, SOD).

### 2.4. Efficacy Criteria

The clinical efficacy of the two groups was compared, and the clinical efficacy of the two groups was evaluated according to the relevant standards in the “Clinical Research Standards for New Drugs” and divided into markedly effective, effective, and ineffective. Markedly effective: blood pressure dropped to the normal range or DBP decreased by ≥ 10 mmHg or SBP decreased by ≥ 20 mmHg; effective: DBP decreased by < 10 mmHg or SBP decreased by 10–20 mmHg, but blood pressure did not decrease to the normal range; invalid: after treatment, blood pressure did not drop significantly and did not reach the standard of markedly effective and effective. Total effective rate (%) = apparent rate (%) + effective rate (%).

### 2.5. Statistical Processing

The SPSS 26.0 software was used to process the obtained data, and the measurement data were expressed in the form of (mean ± variance). The data comparison was performed by the independent sample *t*-test, and the comparison before and after treatment in the same group was by the paired *t*-test; count data were compared using the chi-square test. All calculated *P* values are two-tailed and *P* > 0.05 was considered significant.

## 3. Results

### 3.1. Comparison of the Clinical Efficacy of the Two Groups

The total effective rates of the patients in the valsartan group and the amlodipine group were 80.0% (32/40) and 85.71% (36/42), respectively, and there was no statistical significance in the chi-square test (*P* > 0.05) (Table 2).

### 3.2. Comparison of Blood Pressure Variability between the Two Groups before and after Treatment

Before treatment, the 24 h mean DBP, SBP, 24HSBP, and DBP coefficient of variation of the two groups were compared, and the difference was not statistically significant (*P* > 0.05). The coefficients of variation were significantly decreased, but there was no significant difference between the two groups (*P* > 0.05) (Table 3).

### 3.3. Changes of Serum Vascular Endothelial Function Indexes and FMD% in the Two Groups before and after Treatment

Before treatment, there was no significant difference in H-FABP, vWF, NO, FMD, and NMD between the two groups (*P* > 0.05). FMD and NMD were higher than those before treatment (*P* > 0.05), and the values of H-FABP, vWF, and NO in the valsartan group were lower than those in the amlodipine group, while the values of FMD and NMD were higher than those in the amlodipine group (*P* > 0.05) (Table 4).

### 3.4. Comparison of Oxidative Stress Indicators before and after Treatment in the Two Groups of Patients

Before treatment, there was no significant difference in MDA, GSH-Px, and SOD values between the two groups (*P* > 0.05). The SOD and GSH-Px values in the valsartan group were higher than those in the amlodipine group, and the difference between the two groups was statistically significant (*P* > 0.05) (Table 5).

## 4. Discussion

Hypertension is on the rise globally and is a major risk factor for cardiovascular mortality worldwide. Hypertension is present in 60–70% of people over the age of 60 and can lead to cardiovascular complications such as stroke, coronary heart disease, and heart failure [1]. The World Health Organization estimates that diagnoses of hypertension will increase by 60% between 2000 and 2025. H-type hypertension refers to a special type of hypertension that is complicated by primary hypertension and homocysteine levels. In China, about 75% of hypertensive patients suffer from hyperhomocysteinemia at the same time [2]. Elevated serum Hhy levels in patients with H-type hypertension can lead to vascular endothelial dysfunction, leading to proliferation of vascular smooth muscle cells and platelet aggregation, further exacerbating the disease. In this study, by comparing the improvement of valsartan and amlodipine on vascular endothelial dysfunction and oxidative stress in elderly patients with H-type hypertension, it was found that both drugs could improve vascular endothelial function and reduce the production of reactive oxygen species. Valsartan was better than amlodipine in improving vascular endothelial dysfunction and oxidative stress levels.

At present, drug treatment strategies are often adopted for elderly patients with H-type hypertension, and valsartan and amlodipine are usually designated as first-line antihypertensive drugs. Valsartan is an oral nonpeptide ARB for the treatment of hypertension that inhibits the type II angiotensin receptor associated with reduced aldosterone secretion. It regulates the renin-angiotensin-aldosterone system by blocking the activation of the angiotensin II AT type 1 receptor, resulting in vasodilation, decreased vasopressin secretion, and decreased aldosterone production and secretion. This causes the arterioles and veins to dilate, resulting in a drop in blood pressure (BP) [3]. Amlodipine is a long-acting calcium ion antagonist that inhibits the flow of calcium into vascular smooth muscle cells through L-type calcium channels, prevents vasoconstriction while improving blood flow, and is more effective in inducing vascular relaxation and lowering blood pressure [4]. Studies have shown that amlodipine can promote the release of vascular endogenous factors and can play a protective function of vascular endothelium. Compared with most antihypertensive drugs, it inhibits calcium ion slow channel transmembrane influx into vascular smooth muscle and myocardium with fewer side effects and a longer half-life [5]. The results of this study showed that after 24 weeks of valsartan or amlodipine treatment, compared with the baseline value, the 24 h mean SBP, SDP, 24HSBP, and DBP variation coefficient of the two groups of patients were significantly decreased, and there was no significant difference between the two groups, which suggested that valsartan and amlodipine have good clinical efficacy in the treatment of elderly H-type hypertension.

Studies have shown that the vascular endothelium regulates vascular tone and structure, and endothelial dysfunction and structural changes may be responsible for the adverse effects of hypertension [6]. Endothelial function is determined by the balance between NO and superoxide production. Endothelial dysfunction is characterized by an imbalance in signaling between endothelial-derived vasodilators (e.g., nitric oxide and prostacyclin) and vasoconstrictors [7]. Bioavailable NO can be scavenged by superoxide, and an important source of superoxide production is NADPH oxidase, which is activated by AT1 receptor stimulation. Therefore, ARBs may improve endothelial dysfunction through this mechanism. NO is a vasodilator, which is produced by vascular endothelial cells and has a strong effect on the dilation of blood vessels [8]. It has been reported that a large number of NO produced in plasma of healthy individuals can regulate the cardiovascular system; whereas, in hypertensive patients, NO secretion is reduced. The endothelium regulates vascular tone by balancing the production of vasodilator molecules such as NO. When the vascular endothelium is damaged, a large amount of oxygen free radicals are released, resulting in a decrease in NO levels, contraction of vascular smooth muscles, and increased blood pressure [9]. vWF is a vasoconstrictor factor produced by vascular endothelial cells, which can make platelets tend to the site of endothelial injury and is a marker of vascular endothelial injury or stress response [10]. This study used FMD to assess endothelial function, which is the gold standard for assessing endothelial dysfunction and a predictor of future cardiovascular events and risk of coronary heart disease [11]. Previous studies have shown that valsartan increases FMD, improves endothelial function, and reduces markers of oxidative stress in hypertensive patients. After 24 weeks of treatment in this study, the H-FABP, vWF, and NO values in both groups decreased; the valsartan group decreased more significantly, while the foot-and-mouth disease and NMD in both groups increased; and the valsartan group increased. The higher is more significant. The difference between the two groups is statistically significant (*P* > 0.05). The results indicated that the improvement degree of each index of vascular endothelial function in the valsartan group was better than that in the amlodipine group, suggesting that the effect of valsartan in improving the vascular endothelial dysfunction in patients was more significant, and the ideal therapeutic effect could be achieved.

Oxidative stress is defined as the excess production of reactive oxygen species (ROS) in the context of a decrease in antioxidant species, is characterized by an imbalance between ROS overproduction and antioxidant defenses, and is associated with the aging process [12]. Sustained elevation of inflammatory mediators during aging leads to chronic overproduction of ROS, whose overproduction and reduced antioxidant defenses lead to oxidative stress [13]. The increasing attack of ROS and/or the decline of antioxidants, especially glutathione peroxidase, leads to accumulation of cellular damage. There is increasing evidence that the link between oxidative stress and hypertension appears to be endothelial dysfunction. MDA, GSH-Px, and SOD are the main markers of oxidative stress, which are of great value in evaluating the treatment and prognosis of hypertensive patients. MDA is a metabolite of oxygen free radicals and lipid oxidation, which can cause oxidative stress and can reflect the degree of lipid peroxidation and cell damage [14]. It is known to further inhibit the mitochondrial electron transport system and oxidize sulfhydryl groups in proteins, thereby altering their function or disrupting signal transduction pathways. Studies have found that MDA levels in hypertensive patients are higher than those in normotensive patients. As antioxidant enzymes, SOD and GSH-Px are the first lines of defense of cells against oxidative damage [15]. SOD converts superoxide anion to H_2_O_2_, which is a substrate for GSH-Px. When encountering and reacting with glutathione, GSH-Px reduces both H_2_O_2_ and organic hydroperoxides [16]. Both can be used as markers reflecting the body's antioxidant capacity. In a study comparing valsartan and amlodipine in hypertensive patients with left ventricular hypertrophy, ROS produced by monocytes was reduced in the valsartan group but not in the amlodipine group. A study on the effects of valsartan and amlodipine on endothelial function and oxidative stress in patients with essential hypertension also showed a reduction in markers of oxidative stress after 1 year of treatment with valsartan but not amlodipine. Another study on the effects of amlodipine and valsartan on hemodialysis in patients with end-stage renal disease showed that oxidative stress was reduced in both groups. Kim et al. [17] showed that valsartan and amlodipine can reduce oxidative stress indicators in hypertensive patients with type 2 diabetes mellitus. In this study, the levels of MDA in the two groups were lower than those before treatment, the levels of SOD and GSH-Px were higher than those before treatment, and the values of SOD and GSH-Px in the valsartan group were higher than those in the amlodipine group, while the MDA values were lower in the amlodipine group, and the oxidative stress indicators in both groups were improved, but the improvement of the oxidative stress indicators in the valsartan group was better than that in the amlodipine group, suggesting that valsartan alleviates the elderly oxidative stress injury is more effective in hypertensive patients.

In conclusion, valsartan and amlodipine can reduce blood pressure, improve vascular endothelial function, and inhibit oxidative stress in elderly H-type hypertension patients. Furthermore, valsartan has a more significant effect on improving vascular endothelial dysfunction and oxidative stress in elderly patients with H-type hypertension. However, this study has certain limitations, such as the small number of subjects included and the different clinical characteristics of the included patients. Therefore, more long-term follow-up and large multicenter clinical trials are still needed to confirm the improvement of endothelial dysfunction and the prevention of cardiovascular events.

## Figures and Tables

**Table 1:** Comparison of general clinical data of the two groups of patients.

Index	Valsartan group (*n* = 40)	Amlodipine group (*n* = 42)	*t/χ * ^*2*^	*P* value
Old (year, *x̅* ± *s*)	70.78 ± 7.05	69.88 ± 6.92	0.583	0.561
Female (*n*, %)	25 (62.5)	25 (59.52)	0.076	0.782
Smoking history (*n*, %)	14 (35.0)	11 (26.19)	0.750	0.386
History of alcohol intake (*n*, %)	7 (17.5)	9 (21.43)	0.201	0.654
BMI (kg/m^2^, *x̅* ± *s*)	24.85 ± 3.17	24.69 ± 2.80	0.242	0.809
Average disease duration (year, %)	5.94 ± 2.28	5.76 ± 2.31	0.355	0.724
Average SBP (mmHg, *x̅* ± *s*)	165.85 ± 18.86	169.98 ± 16.12	1.068	0.289
Average DBP (mmHg, x̅ ± s)	91.53 ± 14.55	94.71 ± 14.06	1.006	0..317
Hypertension classification (*n*, %)				
Grade I	25 (62.5)	21 (50.0)	0.254	1.300
Grade II	9 (22.5)	12 (28.57)	0.529	0.396
Grade III	6 (15.0)	9 (21.43)	0.452	0.567
Laboratory metrics (*x̅* ± *s*)				
TC (mmol/L)	4.49 ± 1.21	4.62 ± 1.08	0.514	0.608
TG (mmol/L)	1.46 ± 0.40	1.54 ± 0.39	0.917	0.362
LDL-C (mmol/L)	2.84 ± 0.93	2.71 ± 0.77	0.691	0.492
HDL-C (mmol/L)	1.02 ± 0.20	1.07 ± 0.26	0.973	0.334
Plasma Hcy (*µ*mol/L)	18.10 ± 5.85	19.15 ± 6.90	0.742	0.461
FBP (mmol/L)	4.94 ± 2.31	5.01 ± 2.48	0.132	0.895

DBP, diastolic blood pressure; SBP, systolic blood pressure; TC, total cholesterol; TG, triglyceride; LDL-C, low-density lipoprotein cholesterol; HDL-C, high-density lipoprotein cholesterol; Hcy, homocysteine; FBP, fasting blood glucose.

**Table 2:** Comparison of clinical efficacy between the two groups of patients (*n*, %).

Group	Number of cases	Markedly effective	Effective	Invalid	In total
Valsartan group	40	17 (42.50)	15 (37.5)	8 (20.0)	32 (80.0)
Amlodipine group	42	22 (52.38)	14 (33.33)	6 (14.29)	36 (85.71)
Z/*χ*^2^	–	0.913	0.492		
*P* value	–	0.634	0.473		

**Table 3:** Comparison of blood pressure variability in the two groups before and after treatment.

Group	Cases	24 h mean SBP (mmHg)		24 h mean DBP (mmHg)		24 h SBP coefficient of variation (%)		24 h DBP coefficient of variation (%)	
		Baseline value	After 24 weeks of treatment	Baseline value	After 24 weeks of treatment	Baseline value	After 24 weeks of treatment	Baseline value	After 24 weeks of treatment
Valsartan group	40	164.85 ± 17.34	143.57 ± 9.66	93.26 ± 7.89	81.30 ± 6.23	16.37 ± 3.22	15.20 ± 2.39	13.49 ± 2.65	11.20 ± 2.04
Amlodipine group	42	171.79 ± 15.80	145.50 ± 8.90	91.75 ± 7.34	80.45 ± 6.19	16.15 ± 3.28	14.58 ± 2.41	13.92 ± 2.37	11.89 ± 2.11
*t* value	–	1.896	0.942	0.898	0.620	0.306	1.169	0.775	1.504
*P* value	–	0.062	0.349	0.372	0.537	0.760	0.246	0.440	0.136

SBP, systolic blood pressure; DBP, diastolic blood pressure.

**Table 4:** Comparison of changes in serum endothelial function indexes and FMD% between the two groups before and after treatment (*x̅* ± *s*).

Group	Cases	H-FABP (ng/mL)		vWF (%)		NO (*μ*mol/L)		FMD%		NMD%	
		Baseline value	After 24 weeks of treatment	Baseline value	After 24 weeks of treatment	Baseline value	After 24 weeks of treatment	Baseline value	After 24 weeks of treatment	Baseline value	After 24 weeks of treatment
Valsartan group	40	31.10 ± 5.57	19.25 ± 3.82	187.62 ± 47.31	136.54 ± 28.93	44.73 ± 6.24	32.67 ± 4.10	6.25 ± 1.13	9.46 ± 1.32	13.42 ± 4.38	14.20 ± 3.35
Amlodipine group	42	32.76 ± 6.79	24.53 ± 4.31	200.47 ± 54.96	152.38 ± 39.55	43.91 ± 6.05	37.48 ± 5.39	6.33 ± 1.02	7.28 ± 0.91	12.95 ± 3.10	13.05 ± 3.02
*t* value	-	1.207	5.860	1.134	2.061	0.604	4.531	0.337	8.743	0.563	1.634
*P* value	-	0.231	<0.001	0.260	0.043	0.547	<0.001	0.737	<0.001	0.575	0.106

H-FABP, heart fatty acid binding protein; vWF, von Willebrand factor; NO, nitric oxide; FMD, flow-mediated dilation; NMD, nitroglycerin-mediated dilation.

**Table 5:** Comparison of oxidative stress indicators before and after treatment in the two groups (*x̅* ± *s*).

Group	Cases	Serum MDA (pmol/L)		Serum GSH-Px (*μ*g/ml)		Serum SOD (ng/mL)	
		Baseline value	After 24 weeks of treatment	Baseline value	After 24 weeks of treatment	Baseline value	After 24 weeks of treatment
Valsartan group	40	6.21 ± 2.06	5.71 ± 1.78	13.65 ± 2.59	16.85 ± 2.79	154.78 ± 43.54	188.97 ± 45.67
Amlodipine group	42	6.97 ± 2.48	6.55 ± 2.20	14.31 ± 2.47	15.20 ± 2.34	160.29 ± 41.38	167.30 ± 42.76
*t* value	–	1.506	1.895	1.181	2.907	0.588	2.219
*P* value	–	0.136	0.062	0.241	0.005	0.559	0.029

MDA, malondialdehyde; GSH-Px, glutathione peroxidase; SOD, superoxide dismutase.

## Data Availability

The data used and/or analyzed during the current study are available from the corresponding author upon request.
